# Mutual Regulation of Bcl-2 Proteins Independent of the BH3 Domain as Shown by the BH3-Lacking Protein Bcl-x_AK_

**DOI:** 10.1371/journal.pone.0034549

**Published:** 2012-04-10

**Authors:** Michael Plötz, Amir M. Hossini, Bernhard Gillissen, Peter T. Daniel, Eggert Stockfleth, Jürgen Eberle

**Affiliations:** 1 Department of Dermatology and Allergy, Skin Cancer Center, University Medical Center Charité, Berlin, Germany; 2 Department of Hematology, Oncology and Tumor Immunology, University Medical Center Charité, Berlin, Germany; Roswell Park Cancer Institute, United States of America

## Abstract

The BH3 domain of Bcl-2 proteins was regarded as indispensable for apoptosis induction and for mutual regulation of family members. We recently described Bcl-x_AK_, a proapoptotic splice product of the bcl-x gene, which lacks BH3 but encloses BH2, BH4 and a transmembrane domain. It remained however unclear, how Bcl-x_AK_ may trigger apoptosis.

For efficient overexpression, Bcl-x_AK_ was subcloned in an adenoviral vector under Tet-OFF control. The construct resulted in significant apoptosis induction in melanoma and nonmelanoma cell lines with up to 50% apoptotic cells as well as decreased cell proliferation and survival. Disruption of mitochondrial membrane potential, and cytochrome c release clearly indicated activation of the mitochondrial apoptosis pathways. Both Bax and Bak were activated as shown by clustering and conformation analysis. Mitochondrial translocation of Bcl-x_AK_ appeared as an essential and initial step. Bcl-x_AK_ was critically dependent on either Bax or Bak, and apoptosis was abrogated in Bax/Bak double knockout conditions as well by overexpression of Bcl-2 or Bcl-x_L_. A direct interaction with Bcl-2, Bax, Bad, Noxa or Puma was however not seen by immunoprecipitation. Thus besides BH3-mediated interactions, there exists an additional way for mutual regulation of Bcl-2 proteins, which is independent of the BH3. This pathway appears to play a supplementary role also for other proapoptotic family members, and its unraveling may help to overcome therapy resistance in cancer.

## Introduction

Apoptosis is a defined genetic death program that leads to ordered destruction of cellular components while membrane integrity is preserved [1]. It also represents a safeguard mechanism against tumor formation, due to the elimination of altered and mutated cells. Thus, apoptosis resistance is characteristic for tumor cells, and therapeutic strategies aim to overcome this resistance [2].

Two major apoptosis pathways (extrinsic and intrinsic) have been described in detail. Extrinsic pathways are initiated by binding of death ligands (TNF-α, CD95L and TRAIL) to cell surface receptors, leading to the formation of death-inducing signaling complexes, where initiator caspases 8 and 10 are activated [3], [4]. On the other hand, intrinsic/mitochondrial apoptosis pathways are triggered by intracellular signals such as by cellular or DNA damage. Key events are depolarization of the mitochondrial membrane potential (Δψ_m_) and mitochondrial outer membrane permeabilisation (MOMP) resulting in cytochrome c release and subsequent activation of initiator caspase 9 [5]. Initiator caspases cleave and activate downstream effector caspases, which target a large number of death substrates to set apoptosis into work [6], [7].

Mitochondrial activation is critically controlled by the family of pro- and antiapoptotic Bcl-2 proteins [8]. These proteins share homology in four conserved regions termed Bcl-2 homology domains (BH) and in a transmembrane domain (TM). Antiapoptotic proteins as Bcl-2, Bcl-x_L_, Bcl-w, Mcl-1 and Bfl-1/A1 enclose all four BH domains whereas proapoptotic Bcl-2 homologues subdivide in the Bax/Bak group characterized by BH 1–3, and the BH3-only group enclosing several proteins i.e. Bad, Bid, Bik/Nbk, Bim, Noxa and Puma. In present models, Bax and Bak drive MOMP and are neutralized by antiapoptotic family members. The BH3-only proteins contribute to the regulation either as sensitizers through inhibition of antiapoptotic Bcl-2 proteins or as direct activators of Bax and Bak [8], [9].

Mutual regulation and neutralization has been described as based on the formation of heterodimers between Bcl-2 family members. Thus, the BH3 domain of proapoptotic Bcl-2 proteins encloses an amphipathic α helix, which binds to a hydrophobic groove formed by BH1, BH2 and BH3 of antiapoptotic members [10]. In a rheostat model, the balance of pro- and antiapoptotic Bcl-2 proteins determines the fate of a cell [11]. In melanoma, apoptosis deficiency has been attributed to high expression of antiapoptotic Bcl-2 proteins [12], [13].

Alternative splicing further increases the number of the Bcl-2 family members. Thus, the *bcl-x* gene is expressed as a long antiapoptotic form (Bcl-x_L_) and a short proapoptotic form (Bcl-x_S_) [14]. We have recently described Bcl-x_AK_ (atypical killer), a new proapoptotic splice product which encloses BH2, BH4 and TM. It completely lacks the BH3 domain, which has been regarded so far as indispensable for the proapoptotic function [15].

For unraveling the mechanism of Bcl-x_AK_-mediated apoptosis and exploring its possible therapeutic potential, we constructed an adenoviral vector, which mediates its efficient and conditional expression. We show that Bcl-x_AK_ clearly activated the mitochondrial pathway, and its activity was critically controlled by both pro- and anti-apoptotic Bcl-2 proteins, despite the lack of BH3. Thus, a new model is suggested, in which Bcl-x_AK_ acts as an atypical killer to trigger Bax/Bak-dependent apoptosis.

## Materials and Methods

### Cell culture and cell lines

Three representative human melanoma cell lines, SK-Mel-13 [16], Mel-2a and A-375 [17] were investigated. For analyzing the function of Bax and Bak, the prostate carcinoma cell line DU145 (DSMZ, Braunschweig, Germany) and the colon carcinoma cell line HCT116 (ATCC, Maryland, MD, USA) were used.

Parental DU145 cells are deficient for Bax and reveal only moderate expression of Bak. The cells had been reconstituted by EGFP-tagged Bax or Bak, resulting in DU145-EGFP-Bax and DU145-EGFP-Bak, as described previously [18]. HCT116 parental cells express both Bax and Bak. Isogenic sublines with either Bax knockout or Bak knockdown as well as Bax^−^/Bak^−^ double knockdown cells had been kindly provided by B. Vogelstein (John Hopkins Cancer Center, Baltimore) [18]. Subclones of A-375 melanoma cells resulted from stable tansfection of a pIRES-Bcl-2 plasmid (A375-Bcl-2) or the pIRES empty plasmid (A375-Mock), as previously described [13]. The pIRES plasmid originated from Clontech (Palo Alto, California, USA).

Cell lines were cultured at 37°C, 5% CO_2_ in DMEM (Gibco, Karlsruhe, Germany) supplemented with 10% FCS and antibiotics (Biochrom, Berlin, Germany). For caspase inhibition, cells were preincubated for 1 h with 10 µM of the pancaspase inhibitior zVAD-fmk (R&D Systems, Wiesbaden, Germany), which binds the active sites of caspase-like proteases.

### Construction of Bcl-x_AK_ adenovirus

Bcl-x_AK_ full-length cDNA [15] was subcloned into the Ad5 adenoviral vector pAd5-tTA, according to a strategy described previously [19]. In brief, the cDNA was inserted into the TRE-containing pHVAd2 shuttle vector. The resulting TRE-Bcl-x_AK_ expression cassette was then inserted into pAd5-tTA by homologous recombination, thereby replacing the E1 region and creating pAdV-AK DNA (Fig. 1A). This was transfected into HEK293 cells, and adenoviral plaques corresponding to AdV-AK were propagated. Expression of Bcl-x_AK_ after AdV-AK transduction was suppressed by addition of 1 µg/ml doxycycline to the culture medium (OFF condition), whereas omitting doxycycline resulted in promoter induction (ON condition). An adenoviral vector for expression of myc-tagged Bik/Nbk (Ad5-myc-Nkb-tTA=AdV-Nbk), used here as control, had been described previously [19]. A luciferase-encoding adenovirus (Ad5-CMV-Luc) served as mock control for adenovirus transduction and was applied at the same MOI [20].

**Figure 1:** Efficient induction of cell death by Bcl-x_AK_. (A) The structure of the adenoviral construct AdV-AK is shown. The adenoviral E1 region was replaced by the Bcl-x_AK_ cDNA driven by a tetracyclin-responsive promoter (P_TRE_), and the E3 region was replaced by the tetracyclin-controlled transactivator (tTA) driven by a CMV promoter (P_CMV_). The tTA mediates Tet-OFF regulation. Striped boxes indicate the poly(A)+ regions. (B) Bcl-x_AK_ expression as determined by Western blot analysis is shown in melanoma cell lines SK-Mel-13, A-375 and Mel-2a at 48 h after transduction with AdV-AK (MOI=50). Cells had received doxycycline (OFF condition) or were left without (ON condition). Equal protein loading was confirmed by β-actin. (C) Left, examples of cell cycle analysis after PI staining indicating sub-G1 apoptotic cell populations in Mel-2a at 48 h of transduction. Middle panel, detached and rounded cells indicating apoptosis are shown of Mel-2a at 48 h after transduction with AdV-AK under OFF and ON conditions. Right panel, chromatin condensation and nuclear fragmentation were visualized by bisbenzimide (DAPI) staining in Mel-2a at 48 h after AdV-AK transduction (MOI=50). D–F) Time course analyses of apoptosis (D, flow cytometry after PI staining), cytotoxicity (E, LDH release) and cell proliferation (F, WST-1 assay) are shown for SK-Mel-13, A-375 and Mel-2a cells at 24, 48 and 72 h after transduction with AdV-AK (50 MOI, +Dox=Off, −Dox=On). As positive controls for induced cytotoxicity, cell lines were completely lysed by triton X-100 (T=100%) or were treated with doxorubicin (D, 500 nM, 72 h). WST-1 values are expressed as percent of non-treated controls (=100%). (G) For comparison, apoptosis induction (sub-G1 cells) by AdV-Nbk is shown for Mel-2a cells at 24 h, 48 h and 72 h (MOI=50). AdV-Nbk shares the same backbone with AdV-AK. For induction, doxycycline was omitted (On). (H) A time course analysis of Bcl-x_AK_ expression (3–48 h) after AdV-AK transduction and promoter induction is shown for Mel-2a, as determined by Western blot analysis. (I) Cell survival was determined according to calcein staining in Mel-2a cells at 48 h of Bcl-x_AK_ induction. A shift to the left indicates calcein-negative (=non viable) cells. (J) Quantification of the calcein experiment. (D, E, F, G, J) Means and standard deviations of triplicate values of representative experiments are shown. A luciferase-encoding adenovirus (Ad5-CMV-Luc) applied at the same MOI served as mock control (M), for controlling adenovirus transduction. All experiments were performed at least twice, resulting in highly comparable results.

### Apoptosis, cytotoxicity, cell proliferation and viability

For quantification of apoptosis, cell cycle analyses were carried out, and apoptotic cells corresponded to cell populations with hypodiploid nuclei [21]. Therefore, cells were seeded in 24-well plates (50,000 cells per well). After incubation, cells were harvested by trypsinisation, washed with ice-cold phosphate-buffered saline (PBS) and incubated for 1 h with the staining buffer, containing 0.1% sodium citrate, 0.1% triton X-100 and propidiumiodide (PI; 40 µg/ml; Sigma-Aldrich, Taufkirchen, Germany). The DNA content of nuclei was determined by using flow cytometry (FACSCalibur and CellQuest software; Becton Dickinson, Heidelberg, Germany). As a second assay for quantification of apoptosis, a cell death detection ELISA (Roche Diagnostics, Mannheim, Germany) was applied, which detects mono and oligonucleosomes formed in apoptotic cells. Cytotoxicity was determined in parallel by a cytotoxicity detection assay (Roche Diagnostics), which measures LDH activity in culture fluids. As positive controls for induced cytotoxicity, cells were completely lysed by triton X-100 or were treated with doxorubicin (500 nM, 72 h). Protocols for apoptosis ELISA and LDH release were according to the manufacturer with minor modifications [22].

Cell proliferation (as a product of cell number and mitochondrial activity) was quantified according to the cleavage of the water-soluble tetrazolium salt WST by mitochondrial dehydrogenases in viable cells (WST-1 assay, Roche Diagnostics). Cells were seeded in a density of 10,000 per 100 µl in 96-well plates, and treatments started after 24 h. At the time of analysis, WST-1 reagent was added and absorbance (450 nm) was determined in an ELISA reader. Data were reported in percent of non-treated controls. Cell viability at the single cell level was monitored by the life-cell labeling dye calcein-AM. Briefly, 10^5^ cells were incubated with calcein (4 µM; eBioscience, Frankfurt, Germany) in serum-free growth medium (60 min, 37°C). After PBS washing, cell viability was determined by flow cytometry, comparing calcein-stained (viable) and unstained (dead) cells.

For identification of chromatin condensation and nuclear fragmentation in course of apoptosis, cells were harvested by trypsinisation, centrifuged on cytospins and fixed for 30 min in 4% formaldehyde. Cytospins were stained with bisbenzimide (Hoechst-33258; Sigma, Taufkirchen, Germany; 1 µg/ml, 30 min) and examined by fluorescence microscopy. Apoptotic cells were identified by fragmented nuclei or by bright blue-stained nuclei with condensed chromatin. For quantitative evaluation, fields with 100–200 cells were assessed in triplicates.

### Cell transfection

Melanoma cells were seeded in six-well plates with 2×10^5^ cells/well. For transient transfection, cells at a confluence of 50% were washed with serum-free Opti-MEM medium (Life Technologies, Carlsbad, CA, USA), followed by incubation at 37°C in Opti-MEM for 4 h with plasmid DNA (2.5 or 5 µg/ml) and 0.1% DMRIE-C (Life Technologies). Detailed protocols for transient cell transfection had been described previously [22]. Plasmid constructs of pcDNA3 (Invitrogen, Eugene, OR, USA) were used for transient transfection to express full length Bcl-x_L_ and Bcl-x_AK_.

### Mitochondrial membrane potential and ROS

For determination of the mitochondrial membrane potential (Δψ_m_), the fluorescent dye JC-1 (5,5′,6,6′-tetrachloro-1,1′,3,3′-tetraethyl-benzimidazolyl carbocyanine iodide) or the dye TMRM^+^ (Tetramethyl rhodamine methyl ester perchlorate) were used (both from Sigma-Aldrich). Cells were harvested by trypsinisation and stained for 15 min at 37°C with JC-1 (2.5 µM) or TMRM^+^ (1 µM), and changes of Δψ_m_ were determined by flow cytometry.

For measurement of intracellular ROS levels, the fluorescent dye H_2_DCFDA (2′, 7′- dichloro-dihydro-fluorescein-diacetate) was used. Cells were stained for 30 min with 15 µM H2DCFDA (Molecular Probes, Invitrogen), harvested by trypsinisation, resuspended in HBSS buffer (Biochrom, Berlin, Germany) and analyzed by flow cytometry. For ROS scavenging, N-acetyl cysteine (NAC, Sigma-Aldrich) was used in a concentration of 200 µM.

### Assays for Bax/Bak activation

For determination of Bax and Bak clusters indicative for Bax/Bak activation, DU145 cells were used, which had been stably transfected for expression of EGFP-Bax or EGFP-Bak, respectively [18]. Cells were seeded, transduced with AdV-AK (MOI=50) and were cultured for 48 h with or without doxycycline. Bax and Bak clustering was demonstrated by a fluorescence microscope (Olympus BX50, Hamburg, Germany). For semi-quantitative evaluation, at least 500 cells of each condition were assessed.

For analysis of Bax/Bak conformational changes related to activation, primary antibodies specific for Bax/Bak N-terminal domains were applied in flow cytometry (Bax-NT, Upstate, Lake Placid, USA, #06-499; Bak-NT, Merck, Darmstadt, Germany, #AM04). Melanoma cells (10^5^) were harvested by trypsinisation and fixed for 30 min with 4% paraformaldehyde in PBS. Cells were suspended in saponin buffer (1% FCS, 0.1% saponin in PBS) and incubated for 1 h at 4°C in the dark with antibodies Bax-NT (1∶100) or Bak-NT (1∶10). As secondary antibodies, goat anti-rabbit IgG (H+L)-FITC (Jackson Immuno Research, West Grove, USA) and goat anti-mouse IgG (H+L)-FITC (SouthernBiotech, Birmingham, AL, USA) were used. After washing and resuspension, cells were immediately measured by flow cytometry.

### Western blot analysis

Detailed protocols for protein extraction and Western blot analysis had been described previously [22]. As a standard, 10^6^ cells were harvested and dissolved in lysis buffer (150 mM NaCl, 1 mM EDTA, 0.5% SDS, 0.5% Nonidet P-40, 2 mM PMSF, 1 µM leupeptin, 1 µM pepstatin, 10 mM Tris-HCl, pH 7.5). For analysis of cytochrome c and mitochondrial localization of Bcl-2 proteins, cytosolic and mitochondrial cell fractions were separated by a mitochondria/cytosol fractionation kit (Alexis, Grünberg, Germany).

The following primary antibodies were used: procaspase-3 (Cell Signaling, Danvers, MA, USA; rabbit; 1∶1000), cleaved caspase-3 (Cell Signaling; rabbit; 1∶1000), caspase-8 (Cell Signaling; mouse; 1∶1000), caspase-9 (Cell Signaling; rabbit; 1∶1000), Bcl-x_L_ (Santa Cruz, Heidelberg, Germany; mouse; 1∶200), mouse Bcl-2 (Santa Cruz; mouse; 1∶200), human Bcl-2 (Santa Cruz; mouse; 1∶200), Mcl-1 (Santa Cruz; rabbit; 1∶200), Bax (Santa Cruz; rabbit; 1∶200), Bak (Assay Biotechnology, Sunnyvale, CA, USA; rabbit; 1∶500), Bad (Cell Signaling; rabbit; 1∶1000), Puma (Epitomics, Burlingame, CA USA; rabbit; 1∶1000), Noxa (ProSci Incorporated, Poway, CA, USA; rabbit; 1∶500), cytochrome c (BD Biosciences, Heidelberg, Germany; mouse; 1∶1000), c-Myc (Calbiochem, Nottingham, UK; mouse; 1∶500), anti-porin 31 HL (VDAC; Calbiochem; mouse; 1∶5000), Glyceraldehyde 3-phosphate dehydrogenase (GAPDH; Santa Cruz; mouse; 1∶1000), β-actin (Sigma-Aldrich; mouse; 1∶5000). As secondary antibodies, peroxidase-labeled goat anti-rabbit and goat anti-mouse antibodies were used (Dako, Hamburg, Germany; 1∶5000).

### Immunoprecipitation with anti-Myc microbeads

Melanoma cells (10^6^, SK-Mel-13) were transiently transfected with plasmids encoding myc-tagged Bcl-2 proteins (0.1% DMRIE-C, 5 µg/ml plasmid). After 24 h (for Bcl-x_L_ and Bax) or 48 h (for Bcl-x_AK_), cells were harvested, washed with ice-cold PBS and resuspended in 1 ml of pre-cooled lysis buffer (150 mM NaCl, 1% triton X-100, 50 mM Tris-HCl, pH 8). Microbeads covered with monoclonal anti-myc antibodies were given to the lysate for magnetic labelling of the tagged proteins. Beads and bound proteins were captured on flow-through magnetic columns, washed 4× with buffer 1 (150 mM NaCl, 1% NP-40, 0.5% sodium deoxycholate, 0.1% SDS, 50 mM Tris-HCl, pH 8) and washed for another time with 20 mM Tris-HCl (pH 7.5). Proteins were eluted with hot (95°C) elution buffer (50 mM DTT, 1% SDS, 1 mM EDTA, 0.005% bromphenol blue, 10% glycerol, 50 mM Tris-HCl, pH 6.8). No secondary antibodies were needed. The mock control were melanoma cells transiently transfected with an empty pcDNA3 plasmid. The mock control proved that the anti-Myc beads do not result in any non-specific precipitates. Immunoprecipitation of myc-tagged proteins was carried out with the μMACS c-myc-tagged protein isolation kit (Miltenyi Biotec, Bergisch-Gladbach, Germany). Lysates and immunoprecipitates were investigated by Western blot analysis.

## Results

### Delayed but efficient apoptosis induction

For investigating the efficacy and mechanism of Bcl-x_AK_-mediated apoptosis, an adenoviral vector was constructed with the Bcl-x_AK_ full length cDNA under control of a Tet-OFF promoter inserted into the adenoviral E1 region. The tetracycline/doxycycline repressible transactivator tTA was located in the adenoviral E3 region (Fig. 1A). The construct mediated high expression of Bcl-x_AK_ in melanoma cell lines as shown for SK-Mel-13, A-375 and Mel-2a, when doxycycline was omitted (ON condition), whereas addition of doxycycline almost completely abolished Bcl-x_AK_ expression (OFF condition, Fig. 1B).

Significant induction of apoptosis, as determined by counting hypodiploide sub-G_1_ cells, was seen in melanoma cell lines after transduction and promoter activation, whereas doxycyline strongly diminished apoptosis (Fig. 1D, examples shown in 1C left panel). Kinetic analyses revealed a delayed induction of apoptosis in the three cell lines, which increased to 12%–23% at 48 h and to 17%–37% at 72 h after transduction (Fig. 1D). In contrast, other proapoptotic Bcl-2 proteins induced apoptosis already at 24 h, as shown here for the BH3-only protein Bik/Nbk subcloned in the same adenoviral background (Fig. 1G). The delay in apoptosis induction by Bcl-x_AK_ occurred despite its adenovirus-mediated high expression already at 6 h after transduction (Fig. 1H). Comparable results concerning increased DNA fragmentation were obtained by an apoptosis ELISA (data not shown).

In parallel with DNA fragmentation, clearly visible effects indicating apoptosis were evident, as reduced cell numbers, rounded and detached cells (Fig. 1C, middle panel). Chromatin condensation and nuclear fragmentation, typical hallmarks in apoptosis, were seen after bisbenzimide staining (Fig. 1C, right panel). At 48 h after transduction of Bcl-x_AK_, the cell numbers with atypical nuclei increased from 4% (Off) to 33% (On).

LDH release monitoring loss of plasma membrane integrity was determined to exclude early necrotic cell death. Indeed, LDH release was not significant at 48 h, when apoptosis was already induced, and it was less affected at 72 h, as compared to cytotoxicity controls (Fig. 1E). As determined by WST-1 assay, cell proliferation of Mel-2a cells was strongly decreased, reaching a loss of 60% at 72 h (Fig. 1F). Also cell viability, determined by calcein staining, was decreased (38% in Mel-2a at 72 h), as compared to 6% under Off conditions (Fig. 2I, J). Thus, Bcl-x_AK_ triggered delayed but efficient induction of apoptosis in melanoma cells.

**Figure 2:** Activation of caspases and mitochondria. (A) Processing of caspase-3, -8 and -9 is shown in Mel-2a cells at 24 h and at 48 h after transduction with AdV-AK (MOI=50). Expression of Bcl-x_AK_ was switched on in the absence of doxycycline (ON) or shut off with doxycycline (OFF). Equal protein loading (20 µg/lane) was confirmed by GAPDH. The whole experiment was performed twice. (B) Inhibition of apoptosis by preincubation with the pancaspase inhibitor zVAD-fmk (1 h, 10 µM) is shown. SK-Mel-13 cells had been transduced with AdV-AK (MOI=100, 48 h). Means and SDs of triplicate values of a representative experiment (one of two) are shown. (C) Decrease of the mitochondrial membrane potential (Δψ_m_) is shown for Mel-2a cells at 48 h after transduction of AdV-AK, as determined by flow cytometry after JC-1 or TMRM^+^ staining. Cultures with doxycycline (OFF, grey) are compared to cultures grown in the absence of doxycycline (ON, open graphs). The experiment was performed three times, resulting in highly comparable results. (D) ROS levels were determined in Mel-2a cells at 24 h and 48 h after transduction with AdV-AK under ON and OFF conditions (flow cytometry after H_2_DCFDA staining). Below, parallel cultures were pre-treated for 1 h with 200 µM NAC before transduction. (E) Relative DNA-fragmentation rates (apoptosis) at 48 h with or without NAC were determined in parallel. Non-transduced cells (−/+NAC) are shown as additional controls (open bars). Values had been normalized with regard to non-treated controls, set to 1. Means and SDs of triplicate values of a representative experiment are shown (two independent experiments). (F) Expression levels of Bcl-2 proteins, of p53 and Survivin were determined by Western blot analysis in Mel-2a cells at 24 h and 48 h after transduction with AdV-AK (ON and OFF conditions). Equal protein loading (20 µg/lane) was confirmed by GAPDH.

### Activation of caspases and mitochondria through adenovirus-encoded Bcl-x_AK_

Targeting of the caspase cascade was investigated in Mel-2a cells by Western blot analyses for the initiator caspases 8 and 9 as well as for the main effector caspase 3. Under conditions of high adenovirus-mediated expression of Bcl-x_AK_ and strong apoptosis induction, also significant processing of these caspases was evident at 48 h of transduction (Fig. 2A). Underlining the role of caspases, Bcl-x_AK_-induced apoptosis was almost completely blocked by the pancaspase inhibitor zVAD-fmk (10 µM; Fig. 2B).

The effects on mitochondrial proapoptotic pathways were monitored by two distinct mitochondrial membrane potential (Δψ_m_)-dependent dyes. Both JC-1 and TMRM^+^ revealed the same result, namely decrease of Δψ_m_ upon Bcl-x_AK_ expression. Interestingly, loss of Δψ_m_ appeared already at 24 h after AdV-AK transduction, thus proving this as an early step in Bcl-x_AK_ signal transduction, before apoptosis became evident (Fig. 2C). Reactive oxidative species (ROS) are regarded as an additional step in apoptosis regulation. Increased ROS levels were determined by flow cytometry after H_2_DCFDA staining and found in Mel-2a cells at 48 h but not at 24 h after transduction, thus characterizing this step likely as a consequence of apoptosis (Fig. 2D). Thus, increased ROS may further enhance the apoptotic effect, which was proven by pretreatment for 1 h with the antioxidant N-acetyl cysteine (NAC). Neutralization of ROS by NAC (Fig. 3D) resulted in a two-fold decrease of Bcl-x_AK_-induced apoptosis (Fig. 2E).

**Figure 3:** Bcl-x_AK_-mediated apoptosis depends on Bax or Bak. (A, C) Expression of Bax and Bak is shown by Western blot analysis in subclones of HCT116 and DU145, respectively. Equal loading was confirmed by incubation with β-actin. Two independent series of protein extracts revealed largely comparable expression. (B) HCT116 parental cells (Bax^+^/Bak^+^) as well as subclones (Bax^−^/Bak^+^), (Bax^+^/Bak^−^) and (Bax^−^/Bak^−^) were transduced with AdV-AK (MOI=50) and cultured under OFF or ON conditions. Relative DNA fragmentation values (apoptosis ELISA) were normalized according to the values of parental cells under OFF conditions (set to 1). (D) DU145 parental cells (Bax^−^/EGFP-Bak^−^) as well as subclones (Bax^−^/EGFP-Bak^+^) and (EGFP-Bax^+^/EGFP-Bak^−^) were transduced with AdV-AK (MOI=50, 100) and cultured under OFF or ON conditions. The percentages of apoptotic cells (sub-G1 populations) are shown, as determined by flow cytometry at 48 h after transduction. (B, D) Means and SDs of triplicate values of a representative experiment are shown (each two independent experiments). Statistical significance as determined by Student's t-test is indicated by asterisks (*, p<0.05; **, p<0.005), when comparing parental cells and subclones under ON conditions.

Despite the clear involvement of the mitochondrial pathway, levels of other Bcl-2 proteins remained rather stable after transduction with AdV-AK, as shown by Western blot analysis at 24 h and at 48 h for Bcl-2, Mcl-1, Bax, Puma and Noxa. Similarly, there were no significant changes of the levels of p53 or Survivin (Fig. 2F).

### Dependency on Bax and Bak

To address the relation of Bcl-x_AK_-induced cell death to Bax and Bak, we used a HCT116-derived colon carcinoma cell model. This consisted of parental Bax^+^/Bak^+^ cells and sublines with either Bax knockout or Bak knockdown as well as Bax^−^/Bak^−^ double knockdown cells (Fig. 3A). AdV-AK (50 MOI, 48 h) revealed strong apoptosis induction in parental cells, whereas both Bax and Bak single knockdown significantly diminished apoptosis, indicating that both proteins may be engaged by Bcl-x_AK_. In accordance, Bcl-x_AK_-induced apoptosis was completely abrogated in the double knockdown cells (Fig. 3B).

In a complementary approach, a DU145 prostate carcinoma cell model was applied. Parental cells are deficient for Bax and reveal only moderate activity of Bak. They had been reconstituted for either Bax or Bak expression by using EGFP-tagged copies (Fig. 3C). Parental DU145 cells were clearly non-responsive to AdV-AK, possibly indicating an endogeneous non-functional Bak. However, the reconstitution of either Bax or Bak strongly enhanced Bcl-x_AK_-mediated apoptosis, resulting in each case in more than 50% apoptotic cells. This again showed that Bcl-x_AK_ can induce apoptosis via both Bax and Bak (Fig. 3D).

Formation of Bax/Bak clusters has been reported as related to proapoptotic function [23]. For monitoring this step, DU145 cells were used that had been stably transfected with EGFP-Bax and EGFP-Bak, respectively. In agreement with the function of both Bax and Bak, Bcl-x_AK_ expression resulted in visible clustering of both EGFP-Bax and EGFP-Bak at 48 h after transduction. Clustering induced by Bcl-x_AK_ was comparable to the effects of doxorubicin (2 µM, 24 h), used as positive control (Fig. 4A). Evaluations revealed Bax/Bak clusters in 20%–30% of cells, similar to apoptosis inductions at these conditions (Fig. 4B). In course of Bax/Bak activation, conformational changes may lead to exposure of their N-termini. Flow cytometry with N-terminus-specific antibodies (Bax-NT, Bak-NT) showed activation of Bax and Bak in 30% of Mel-2a cells in response to Bcl-x_AK_ expression (Fig. 4C, 4D).

**Figure 4:** Bax and Bak activation after Bcl-x_AK_ overexpression. (A) For investigation of Bax and Bak clustering, DU145 cells stably transfected for expression of EGFP-Bax or EGFP-Bak were transduced with AdV-AK and cultured for 48 h under OFF or ON conditions. Doxorubicin-treated cells (2 µM, 24 h) were used as positive controls. Examples of fluorescence microscope images taken at 48 h after transduction and promoter induction are shown. (B) A quantitative evaluation of Bax and Bak clustering was performed (means and SDs of triplicate values of a representative experiment). A second experiment revealed comparable results. (C) Bax and Bak activation upon Bcl-x_AK_ expression was determined in Mel-2a at 48 after AdV-AK transduction (50 MOI), by flow cytometry after staining with conformation-specific antibodies against Bax and Bak N termini (Bax/Bak NT). The bars indicate the populations counted as positive for activated Bax and Bak, respectively. (D) A quantification of triplicate values (one experiment of two independent) is shown. Transduction with AdV-Nbk (50 MOI) is shown for comparison.

### Abrogation of Bcl-x_AK_-mediated apoptosis by antiapoptotic Bcl-2 proteins

To address the role of antiapoptotic Bcl-2 proteins, A-375 melanoma cells stably transfected for Bcl-2 overexpression (A375-Bcl-2) were applied. These cells were completely protected against the proapoptotic effects of Bcl-x_AK_, whereas mock-transfected cells (A375-Mock) revealed about 30% apoptotic cells at 48 h of transduction with AdV-AK (Fig. 5A). A similar result was obtained after Bcl-x_L_ overexpression. Transient transfection of a Bcl-x_AK_ expression plasmid significantly enhanced apoptosis in SK-Mel-13 melanoma cells at 48 h, whereas the co-transfection of a Bcl-x_L_ expression plasmid almost completely prevented Bcl-x_AK_-induced apoptosis (Fig. 5B). Thus, either one or these antiapoptotic proteins was sufficient to block Bcl-x_AK_-mediated apoptosis. Loss of Δψ_m_ was also seen in A375-Mock, which was completely prevented by Bcl-2 overexpression in A375-Bcl-2 (Fig. 5C).

**Figure 5:** Bcl-2 and Bcl-x_L_ block the proapoptotic effects of Bcl-x_AK_. (A) Subclones of A-375 cells stably transfected with pIRES-Bcl-2 (A375-Bcl-2) or mock-transfected (A375-Mock) were transduced with AdV-AK under OFF or ON conditions. Non-transduced cells (−) were used as additional controls. Numbers of apoptotic cells (sub-G1 cell populations) were determined by flow cytometry after PI staining. (B) SK-Mel-13 melanoma cells were transiently transfected with either Bcl-x_L_ or Bcl-x_AK_ alone or with a combination of both (each 2.5 µg plasmid-DNA). Relative DNA fragmentation values, as determined at 24 h and 48 h after transfection, were calculated with respect to cells that had received only the transfection lipid (white bars). (A, B) Means and SDs of triplicate values of a representative experiment are shown (each two independent experiments). Overexpression of Bcl-2, Bcl-x_L_ and Bcl-x_AK_, as determined by Western blot analyses, is shown in the insets. (C) The mitochondrial membrane potential (Δψ_m_) was determined by flow cytometry after TMRM staining in A375-Mock and in A375-Bcl-2 at 24 h and 48 h. After transduction with AdV-AK, inducible and non inducible conditions were compared (On/Off). The experiment was performed three times, giving comparable results.

### Mitochondrial translocation of Bcl-x_AK_ is not prevented by Bcl-2

Hallmarks in mitochondrial apoptosis pathways are translocation of Bax and release of mitochondrial factors. Significant cytochrome c release was seen in Mel-2a and in A375-Mock at 48 h after AdV-AK transduction (Fig. 6A). Also higher levels of Bax were seen in mitochondrial extracts. In this assay however, Bax translocation and activation is underestimated as some cytosolic contaminations (up to 5%) were still left in mitochondrial fractions seen by the cytosolic marker GAPDH. This may explain the weaker bands of Bax already before induction of Bcl-x_AK_ expression (Fig. 6B).

**Figure 6:** Bcl-2 blocks Bcl-x_AK_-mediated cytochrome c release and Bax translocation. Mel-2a, A375-Mock and A375-Bcl-2 cells were transduced with AdV-AK (MOI=50) and were kept under OFF and ON conditions. At 24 h and 48 h, cytosolic fractions (Cyto) and mitochondrial fractions (Mito) were isolated and analysed by Western blotting. Non-transfected controls (−) are shown as controls. The whole experiment was performed two times, resulting in highly comparable results. (A) Cytosolic extracts were analyzed for showing expression of Bcl-x_AK_ and release of cytochrome c. Mitochondrial extracts serve as positive controls, the mitochondrial protein VDAC ruled out any contaminations of cytosolic extracts with mitochondria, and β-actin served as loading control. (B) Mitochondrial extracts were analyzed for showing mitochondrial translocation of Bcl-2 proteins. Here, cytosolic extracts served as controls, equal protein loading was confirmed by VDAC and the relative purity of mitochondrial extracts was examined by GAPDH. 5% of the total mitochondrial fractions and 2% of the total cytosolic fractions had been loaded on the gels.

The localization of Bcl-x_AK_ itself appeared as an important step. When comparing 24 h with 48 h, the amount of Bcl-x_AK_ in the cytosol significantly decreased at 48 h by 2–3-fold in all three cell lines. Equal loading of cytosolic extracts was proven by β-actin (Fig. 6A). The direct comparison of the mitochondrial extracts at 24 h and 48 h clearly showed almost no Bcl-x_AK_ in Mel-2a and only weak bands in the two A-375 clones at 24 h. The mitochondrial localization of Bcl-x_AK_ however strongly increased at 48 h (Fig. 6B). Simultaneous decrease of Bcl-x_AK_ in the cytosol and its strong increase in mitochondria at 48 h clearly proved mitochondrial translocation of Bcl-x_AK_, which is suggestive as a critical step for induction of apoptosis. Importantly, the mitochondrial translocation of Bcl-x_AK_ was not prevented by Bcl-2, whereas cytochrome c release and Bax translocation were completely blocked (Fig. 6A; B).

### No interaction of Bcl-x_AK_ with other Bcl-2 family members

For investigating whether Bcl-x_AK_ might directly interact with other Bcl-2 proteins, SK-Mel-13 melanoma cells were transiently transfected with myc-tagged copies of Bcl-x_AK_, Bcl-x_L_ or Bax. Following immunoprecipitation with anti-Myc microbeads, binding of Bcl-2, Bax, Bad, Noxa and Puma was investigated by Western blotting. Mock transfected cells were used as controls and ruled out non-specific precipitations by the microbeads. On the other hand, Myc-tagged proteins were efficiently immunoprecipitated, as seen in the pellet (P) fractions after incubation with the Myc antibody (Fig. 7A, panels 1–3).

**Figure 7:** Co-immunoprecipitation analyses of Bcl-x_AK_ with Bcl-2 family members. (A) SK-Mel-13 melanoma cells were transiently transfected with each 5 µg of pcDNA3 plasmids encoding Bcl-x_L_, Bcl-x_AK_, Bax or empty vector (Mock). Cells lysates were immunoprecipitated with microbeads covered with anti-Myc antibody, and immunoprecipitates were analysed by Western blotting. Non-bound supernatants (S) were compared with the immunoprecipitated pellet fractions (P). Antibodies for immunodetection: anti- Myc, Bcl-2, Bax and Bad. The complete experiment was performed two times, which both gave the same result. (B) A model for apoptosis induction by Bcl-x_AK_ is suggested. It is based on mitochondrial translocation of Bcl-x_AK_ and activation of Bax/Bak. Bcl-2/Bcl-x_L_ prevent Bax/Bak activation but not Bcl-x_AK_ translocation. BH3-only proteins may mediate a BH3 domain-dependent pathway via inactivation of antiapoptotic Bcl-2 proteins and may also drive a BH3-independent pathway analogous to Bcl-x_AK_ (see discussion part).

The binding analyses revealed characteristic interactions, thus proving the reliability of the assay. Thus binding of Bcl-2 to myc-Bax, binding of Bax to myc-Bcl-x_L_ and myc-Bax as well as binding of Bad to myc-Bcl-x_L_ were seen (Fig. 7A). Apoptosis, monitored in parallel, was induced by myc-Bax and myc-Bcl-x_AK_, whereas myc-Bcl-x_L_ diminished basal apoptotic rates, thus providing a proof on the function of the transfected proteins (data not shown). However, no direct interactions of the five representatives of the Bcl-2 family were seen with Bcl-x_AK_ (Fig. 7A), thus suggesting that Bcl-x_AK_ displays its activation of Bax and Bak in an indirect way via a not yet defined step. In this pathway Bcl-x_AK_ and antiapoptotic family members act independent of each other on Bax and Bak (Fig. 7B).

## Discussion

Pro- and antiapoptotic Bcl-2 proteins are critically involved in apoptosis regulation by controlling mitochondrial cell death pathways [5]. Their already high number is further increased by differential splicing, leading to an enhanced complexity. Thus, up to 10 splice products have been reported for the *bim* gene, of which Bim_S_, Bim_L_ and Bim_EL_ have been characterized. Also eight splice products with different domain structures have been reported for the *bax* gene, of which Bax-α is best characterized [24], [25]. Another example is given by the *bcl-x* gene, which is expressed in four reported isoforms with different activities. Besides Bcl-x_L_ (long), antiapoptotic functions have also been reported for Bcl-x_ES_ (extra short) [26], [27]. In contrast, Bcl-x_S_ (short) and Bcl-x_AK_ (atypical killer) exert proapoptotic functions [14], [15]. Alternative splicing is a target of specific regulations. Thus, the switch from Bcl-x_L_ to Bcl-x_S_ in response to genotoxic stress was related to an ATM/CHK2/p53-dependent pathway [28]. The pathway, which triggers Bcl-x_AK_ expression, is not yet defined.

Bcl-2 proteins are categorized in three subfamilies according to different domain structures, enclosing antiapoptotic proteins (BH 1–4), the Bax/Bak group (BH 1–3) and BH3-only proteins [9]. The *bcl-x* splice products, however, reveal unique structures. Thus, Bcl-x_S_ encloses BH3 and BH4 [24], whereas Bcl-x_AK_ encloses BH2 and BH4 [15]. Despite the BH3 domain has been regarded as indispensible for proapoptotic functions [12], we had previously categorized Bcl-x_AK_ as proapoptotic based on a moderate induction of apoptosis in melanoma cells (two-fold), after plasmid transfection [15]. For unraveling Bcl-x_AK_-mediated pathways, we have constructed an adenoviral vector, which drives its high and conditional expression under Tet-OFF control. With this efficient expression system, Bcl-x_AK_ induced apoptosis in up to 40% of melanoma and in 50% of non-melanoma cells. In its efficacy, Bcl-x_AK_ was comparable to the BH3-only protein Bik/Nbk, which was available in the same adenoviral backbone [19].

Under AdV-AK-mediated high expression of Bcl-x_AK_, significant caspase activation became evident, in contrast to previous findings under moderate expression of Bcl-x_AK_ [15]. Thus, caspase activation by Bcl-x_AK_ in melanoma cells appeared as dependent on its expression level. Initiator caspases of both extrinsic and intrinsic pathways (caspase-8, and −9) were cleaved. However, caspase-8 may also be activated downstream of caspase-3 in a described amplification loop [29], which is suggestive for Bcl-x_AK_.

Bcl-2 family proteins are particularly involved in the control of mitochondrial apoptosis pathways, which can be induced by overexpression of BH3-only proteins as well as by overexpression of Bax or Bak [18], [30], [31]. Also, Bcl-x_AK_ resulted in significant decrease of mitochondrial membrane potential and in cytochrome c release, thus clearly indicating parallels to other proapoptotic Bcl-2 proteins. Although Bax/Bak-independent mechanisms were also discussed [32], mitochondrial activation is mainly related to Bax or Bak function [9]. Here again, Bcl-x_AK_ revealed typical characteristics of proapoptotic Bcl-2 proteins, namely a strong dependency on either Bax or Bak. Both proteins share a similar structure and related functions [33]. Some proapoptotic Bcl-2 proteins show preference for activating either Bax or Bak, as Bik/Nbk and tBid go via Bax [9], [18] and Bcl-x_S_ goes via Bak [34]. For Bcl-x_AK_, however, Bak expression could compensate for loss of Bax and vice versa, and apoptosis induction was abolished only in Bax/Bak double deficient cells. This suggests that Bcl-x_AK_ may may drive more general changes at the mitochondrial membrane rather than selectively targeting a specific protein.

Importantly, after transduction all melanoma cells were responsive to Bcl-x_AK_, as the whole cell population showed reduced Δψm, increased ROS as well as activated Bax and Bak. However, certain thresholds may prevent full apoptosis induction in the majority of cells. This may be related to the activity of antiapoptotic Bcl-2 family members, which may block Bax and Bak. Thus, overexpression of Bcl-2 abrogated apoptosis induced in melanoma cells by Bik/Nbk [35], [36], and Bcl-x_L_ inhibited Bax-induced apoptosis in mouse embryonic fibroblasts [37]. These antiapoptotic activities had been described as dependent on BH3-mediated heterodimerization. However, also the proapoptotic effects of Bcl-x_AK_ were completely inhibited by Bcl-2 or Bcl-x_L_. This may depend on the inhibition of Bax and Bak by the antiapoptotic proteins, rather than on direct inhibition of Bcl-x_AK_. In agreement, Bcl-2 could not prevent Bcl-x_AK_ mitochondrial translocation.

Highly characteristic for Bcl-x_AK_-induced apoptosis was a time delay of 48 h, whereas other Bcl-2 proteins as Bik/Nbk and Bcl-x_S_ induced apoptosis in melanoma cells already at 24 h [35], [36]. In general, proapoptotic signaling as mutual regulation of Bcl-2 proteins, cytochrome c release and caspase activation are rather quick cellular events [38]. The time delay of Bcl-x_AK_ in contrast to other proapoptotic Bcl-2 proteins is indicative for an indirect mechanism enclosing a time-consuming step. No relation was seen to the expression of other Bcl-2 proteins. Rather, Bcl-x_AK_ mitochondrial localization appeared as a critical step, and membrane transport may play a regulatory role therein. Whereas Bcl-x_AK_ was cytosolic at 24 h, it translocated to mitochondria at 48 h, when apoptosis was induced. Also other proapoptotic Bcl-2 proteins have to translocate to mitochondria to exert their proapoptotic activities, as shown for tBid and Bax [5], [39]. Thus, apoptosis by Bcl-x_AK_ appeared as tightly linked to its presence in mitochondria, where it resulted in Bax and Bak activation.

An interesting finding was that loss of Δψ_m_ preceded translocation of Bcl-x_AK_ and MOMP. The relation between Δψ_m_ and MOMP is still a matter of discussion; one effect may precede the other or they may even occur independently of each other [40], [41]. Loss of Δψm may result from uncoupling of the mitochondrial electron transport chain which may lead to Bax and Bak oligomerization [42]. Mitochondrial dynamics appears as another important level, which may be influenced by Bcl-x_AK_ overexpression. Mitochondrial dynamics may contribute to the control of MOMP, which is further dependent on Bax [43]. Formation of large Bax/Bak clusters has been suggested, which may translocate to mitochondrial constriction sites, to drive MOMP [23]. Clustering of Bax and Bak was clearly induced in response to Bcl-x_AK_, thus further relations to mitochondrial fission and fusion may be expected.

For BH3-only proteins, different mechanisms have been suggested to explain their proapoptotic activities. In the neutralization/displacement model, BH3-only proteins bind antiapoptotic family members, to release Bax or Bak [5]. This activity is based on BH3, which binds to the hydrophobic groove of antiapoptotic Bcl-2 proteins [44]. According to a second model, BH3-only proteins may also directly bind and activate Bax or Bak, which has been shown for tBid, Bim and Puma [38], [45], [46]. This activity is also regarded as BH3-dependent. Thus, direct, although week binding of Bim to Bax has been shown, which was abrogated by the replacement of the Bim BH3 [30]. Also peptides of the BH3 domains of Bid, Bim and Puma were able to drive direct activation of Bax [45]. Both ways of apoptosis induction can not apply to Bcl-x_AK_, due to its lack of BH3.

A third way of apoptosis induction has been recently suggested. It is explained by a general remodelling of the mitochondrial outer membrane, and it was also seen after intercalation of BH3-only proteins, which resulted in Bax activation [47]. Of note, this proapoptotic activity appeared as independent of the BH3 domain. Thus for the BH3-only protein Bnip3, the transmembrane domain (TM) has been proven as essential for its proapoptotic activity, whereas BH3 could be mutated without major effect on apoptosis induction [48]. Also for Bim_S_, deletion or point mutation of its BH3 on one hand prevented the interaction with Bcl-2 and Bax but remained largely without effect on apoptosis induction. Bim_S_ mutants still localized to mitochondria, suggesting that this was the critical step, and indeed, when the TM was deleted, the proapoptotic activity was lost [49]. Also for Bcl-x_AK_, mitochondrial translocation appeared as the critical step. A deletion analysis for Bcl-x_AK_ may become particularly helpful for identification of proapoptotic domain(s) independent of BH3, as overlapping functions with BH3 are here excluded.

Thus, the characterization of Bcl-x_AK_ strongly supports speculations on proapoptotic pathways that are mediated by Bcl-2 proteins but act independent of the BH3 domain. These pathways are nevertheless critically dependent on Bax and Bak as well as on antiapoptotic Bcl-2 family members. As shown here for melanoma, colon and prostate carcinoma cells, activation of these pathways can be effective in cancer cells. Bcl-2 proteins are of critical importance for therapy resistance in cancer, as particularly seen in melanoma [2]. Thus, new pathways for regulating Bcl-2 protein activity are of particular interest and may become useful for targeting so far therapy-refractory tumors, such as melanoma.
